The article "Effects of Shenkang Injection Combined with Jinshuibao on Early Diabetic Nephropathy and Effects on Coagulation Fibrinolysis System and Urinary Protein" was retracted in 2023. Reasons: signs of a paper mill; suspected computer-generated content; unreliable results or conclusions; concerns about the data.

# Effects of Shenkang Injection Combined with Jinshuibao on Early Diabetic Nephropathy and Effects on Coagulation Fibrinolysis System and Urinary Protein

**DOI:** 10.1155/2022/3958049

**Published:** 2022-10-11

**Authors:** Jianhua Zhu, Tingting Yang, Jie Luo, Mian Wei, Hanyu Li, Yue Qi, Jiali He, Min Chen

**Affiliations:** Department of Nephrology, Chengdu Hospital of Integrated Traditional Chinese and Western Medicine, Chengdu, Sichuan 610000, China

## Abstract

**Purpose:**

To explore the effect of Shenkang injection (SKI) combined with Jinshuibao for early diabetic nephropathy (DN) and its effect on the coagulation fibrinolysis system and urinary protein.

**Methods:**

136 patients with early DN admitted to our hospital from March 2018 to October 2019 were divided into the observation group (*n* = 68) and the control group (*n* = 68) randomly. On the basis of the conventional treatment, the control group was treated with SKI, and the observation group was treated with SKI and Jinshuibao. Two weeks later, the therapeutic effects of the 2 groups were compared. The prothrombin time (PT), activated partial thromboplastin time (APTT), thrombin time (TT), fibrinogen (FIB), tissue plasminogen activator (*t*-PA), plasminogen activator inhibitor-1 (PAI-1), and D-dimer (D-D) were observed and compared before and after the treatment. 24 hour urine total protein (24 h-UTP), urine albumin excretion rate (UAER), and urine *β*_2_ microglobulin (*β*_2_-MG) were measured and compared before and after the treatment. Adverse reactions in the two groups were recorded during the treatment.

**Results:**

The effective rate of the observation group after treatment was 92.65% higher than the control group 79.41%. the difference was statistically significant (*P* < 0.05). The levels of PT, APTT, TT, FIB, PAI-1, and D-D in the two groups after treatment were lower, and t-PA levels after treatment were higher than those before, and all of the above indicators were significantly changed in the observation group than in the control group. The difference was statistically significant (*P* < 0.05). The 24 h-UTP, UAER, and *β*_2_-MG in the two groups after treatment were lower than those before, and all of the above indicators were significantly changed in the observation group than in the control group. The difference was statistically significant (*P* < 0.05). There was no statistically significant difference during the treatment for 2 groups in terms of adverse reactions. The difference was statistically significant (*P* > 0.05).

**Conclusion:**

SKI combined with Jinshuibao has a significant effect in the treatment of early DN, which can reduce the risk of hyperfunction of coagulation and fibrinolysis system, further reduce the content of urine protein, and delay the process of DN.

The article "Effects of Shenkang Injection Combined with Jinshuibao on Early Diabetic Nephropathy and Effects on Coagulation Fibrinolysis System and Urinary Protein" was retracted in 2023. Reasons: signs of a paper mill; suspected computer-generated content; unreliable results or conclusions; concerns about the data.

## 1. Introduction

Diabetes mellitus (DM) is a group of chronic metabolic diseases characterised by high blood sugar. Persistent hyperglycaemia directly causes chronic damage to various tissues and organs in the body, such as the retina, heart, kidneys, and vascular nerves, leading to a series of chronic complications of DM [1, 2]. Nephropathy is one of the serious microvascular complications of DM, an important cause of chronic renal insufficiency and also an important cause of disability and death in DM patients [3]. Patients with early diabetic nephropathy (DN) usually present with trace proteinuria, oedema, and few clinical symptoms. At the same time, microcirculatory disorders can occur due to abnormal blood glucose and lipid metabolism, which can lead to changes in the coagulation and fibrinolytic systems such as hypercoagulability and fibrinolytic abnormalities. It is now believed that effective intervention in the early stages of DN can delay or even reverse further deterioration of renal function.

The pathogenesis of DN involves hemodynamic abnormalities, hemorheological changes, glomerular basement membrane thickening (biochemical metabolic disorders), genetic susceptibility, and other factors [4–7]. Shenkang injection (SKI) is a new class II Chinese medicine consisting of four Chinese herbs, namely rhubarb, *Astragalus* membranaceus, *Salvia miltiorrhiza,* and safflower, which are effective in dredging the bowels and purging turbidity, supplementing qi, and activating blood circulation. In recent decades, SKI has been most commonly used in clinics to treat kidney-related diseases. It can inhibit the proliferation of glomerular mesangial cells (MC), reduce the accumulation of extracellular matrix (ECM), and delay glomerular sclerosis so as to improve the renal function of patients and delay the progression of kidney disease [8]. The curative effect is accurate. At the same time, a large number of studies have also confirmed that SKI can improve cardiorenal syndrome, hepatorenal syndrome, COPD, and other diseases. Jinshuibao is a kind of Cordyceps sinensis extract, which has the effects of being antibacterial, anti-inflammatory, reducing serum cholesterol, triglycerides, and lipid peroxides, increasing blood supply to the myocardium and brain, and nourishing the lungs and kidneys [9]. This study investigated the efficacy of SKI combined with Jinshuibao in the treatment of early DN and its effect on the coagulation fibrinolysis system and urinary protein.

## 2. Materials and Methods

### 2.1. Research Object

136 patients with early DN admitted to our hospital from March 2018 to October 2019 were divided into the observation group (*n* = 68) and the control group (*n* = 68) randomly. In the control group, there were 37 males and 31 females, with a mean age of 52.1 ± 3.9 years and a mean duration of illness of 5.9 ± 3.5 years; in the observation group, there were 35 males and 33 females, with a mean age of 51.3 ± 3.6 years and a mean duration of illness of 6.4 ± 2.7 years. All the above basic data were compared, and the differences were not statistically significant (*P* > 0.05) and comparable.

The article "Effects of Shenkang Injection Combined with Jinshuibao on Early Diabetic Nephropathy and Effects on Coagulation Fibrinolysis System and Urinary Protein" was retracted in 2023. Reasons: signs of a paper mill; suspected computer-generated content; unreliable results or conclusions; concerns about the data.

### 2.2. Diagnostic Criteria

#### 2.2.1. DM Diagnostic Criteria

Referring to the 2004 Chinese guidelines for the prevention and treatment of diabetes [10], with clinical signs of DM + determination of plasma glucose ≥11.1 mmol/L (200 mg/dL); determination of fasting blood glucose (FBG) ≥7.0 mmol/L (126 mg/dL); 2 hours after ƒOGTT test, plasma glucose ≥11.1 mmol/l (200 mg/dl). If any of the above three items were met, it could be used as a diagnostic basis. In the absence of hyperglycaemic crisis, a single blood glucose level up to the diagnostic criteria for DM must be rechecked at a later date for verification.

#### 2.2.2. DN Staging Criteria

Referring to the internationally accepted Mogensen staging [11], i.e., DN stage III: 2 positive urine tests for microalbumin (MA) [urine albumin to creatinine ratio (ACR) 2.5∼30.0 mg/mmol (men) and 3.5∼30.0 mg/mmol (women) at any time point]; or 24 hour urine microalbumin (U-MA) quantification of 20∼200 mg/L; or urine albumin excretion rate (UAER) 20∼200 *μ*g/min (30∼300 mg/24 h); urine routine protein negative, 24 hour urine total protein (24 h-UTP) <0.5 g; and excluded other factors causing increased urine protein.

### 2.3. Inclusion Criteria

(1) Meeting the above diagnostic criteria for DM and the Mogensen staging criteria for DN stage III; (2) those who volunteered to participate in this study; and (3) those who were not taking ACEI or ARB class antihypertensive drugs.

### 2.4. Exclusion Criteria

(1) Persons with chronic glomerulonephritis, nephrotic syndrome, urinary tract infections, urinary stones, and other urological disorders; (2) persons with primary renal insufficiency or renal artery stenosis; (3) persons with elevated blood potassium or abnormal blood creatinine; (4) persons with diabetic ketosis, ketoacidosis or co-infections, and other systemic diseases; (5) patients with cardiovascular and cerebrovascular diseases and disorders of blood clotting; (6) women during pregnancy and breastfeeding; (7) persons who had recently taken antiplatelet or anticoagulant medication or were allergic to the study medication; and (8) persons who had interrupted treatment before completing the prescribed course of treatment, whose efficacy could not be judged or whose data were incomplete.

The article "Effects of Shenkang Injection Combined with Jinshuibao on Early Diabetic Nephropathy and Effects on Coagulation Fibrinolysis System and Urinary Protein" was retracted in 2023. Reasons: signs of a paper mill; suspected computer-generated content; unreliable results or conclusions; concerns about the data.

### 2.5. Research Methods

Both groups were given oral hypoglycaemic drugs or subcutaneous insulin for blood glucose control, a diabetic diet, and moderate exercise as a general treatment, depending on the condition of the patients. In the control group, SKI (Xi'an Century Shengkang Pharmaceutical Co., Ltd., State Drug Administration Z20040110) was administered 100 ml + 0.9% sodium chloride injection, 250 ml intravenous drip, 1 time/d. In the observation group, Jinshuibao (Jiangxi Jimin Kexin Jinshuibao Pharmaceutical Co., Ltd., State Drug Administration Z10890003) was added on top of the control group for oral administration, 3 capsules/time, 3 times/d. Both groups were treated continuously for 2 weeks.

### 2.6. Observation Indicators

Efficacy was determined after 2 weeks of treatment [12]. Apparently cured: significant improvement in symptoms such as oedema, significant improvement in all urine protein-related indicators, and control and cessation of the progression of the disease; improved: symptoms such as oedema had improved, all urine protein-related indicators had improved, and renal disease was progressing slowly; invalid: symptoms such as oedema and proteinuria remain and did not improve or the kidneys deteriorate further. Total effective rate = (number of apparently cured cases + number of improved cases)/total number of cases × 100%.

Then, 10 ml of the fasting venous blood was collected from patients before and 2 weeks after treatment, centrifuged, and the serum was prepared. Prothrombin time (PT), activated partial thromboplastin time (APTT), thrombin time (TT), and fibrinogen (FIB) by the coagulation method and tissue plasminogen activator (t-PA), plasminogen activator inhibitor-1 (PAI-1), and D-dimer (D-D) by the ELISA method.

Patients' urine were collected 24 h before treatment and 24 h after 2 weeks of treatment, and 10 ml was taken after thorough mixing for examination. The 24 h-UTP was measured by urine protein precipitation and the biuret method, and urine *β*_2_ microglobulin (*β*_2_-MG) and MA concentrations were measured by immunoturbidimetric assay and UAER was calculated.

The adverse reactions of patients in both the groups were observed during the treatment period.

### 2.7. Statistical Methods

The SPSS22.0 software was applied for processing and the count data were expressed as rate (%) using the *χ*^*2*^ test. The measurement data were expressed as mean ± standard deviation ($\bar{x}\pm s$) and the *t*-test was used for two-way comparison between groups. The test level was *α* = 0.05 and *P* < 0.05 was considered a statistically significant difference.

The article "Effects of Shenkang Injection Combined with Jinshuibao on Early Diabetic Nephropathy and Effects on Coagulation Fibrinolysis System and Urinary Protein" was retracted in 2023. Reasons: signs of a paper mill; suspected computer-generated content; unreliable results or conclusions; concerns about the data.

## 3. Results

### 3.1. Comparison of Post-Treatment Outcomes for 2 Groups

As shown in Table 1, after treatment, the effective rate of the observation group 92.65% was higher than the control group 79.41%, the difference was statistically significant (*P* < 0.05).

### 3.2. Comparison of Coagulation and Fibrinolytic Parameters for 2 Groups

As shown in Figure 1, before treatment, there was no significant difference in all coagulation and fibrinolytic parameters for 2 groups (*P* > 0.05); after treatment, the levels of PT, APTT, TT, FIB, PAI-1, and D-D in the two groups were lower and *t*-PA levels was higher than those before treatment, and the levels of PT, APTT, TT, FIB, PAI-1, and D-D in the observation group were lower, and the levels of t-PA were higher in the observation group than those in the control group. The difference was statistically significant (*P* < 0.05).

### 3.3. Comparison of Urine Protein Indicators for 2 Groups

As shown in Figure 2, before treatment, there was no significant difference in the comparison of all urine protein indicators for the 2 groups (*P* > 0.05); after treatment, 24 h-UTP, UAER, and *β*_2_-MG in the two groups were lower than those before treatment, and 24 h-UTP, UAER, and *β*_2_-MG in the observation group were lower than those in the control group; the difference was statistically significant (*P* < 0.05).

### 3.4. Comparison of Adverse Reactions for 2 Groups

During the treatment period, there were 2 cases of nausea, 1 case of vomiting, and 1 case of dizziness in the control group, for a total of 4 cases, with an incidence of 5.88% (4/68); 2 cases of nausea, 2 cases of dizziness, and 2 cases of abdominal distension in the observation group, for a total of 6 cases, with an incidence of 8.82% (6/68). Comparison of adverse reactions for 2 groups revealed no statistically significant difference (*P* > 0.05).

## 4. Discussion

DN is a serious group of microvascular complications of DM. Its pathogenesis is very complex, including microcirculation disorders caused by abnormal glucose and lipid metabolism, activation of the RASS system, accumulation of advanced glycoprotein products, tissue oxidative stress response, and abnormal expression of the coagulation and fibrinolysis systems [13]. Early DN is mostly manifested by a high glomerular filtration rate, increased renal volume, thickened basement membrane, microalbuminuria, edema, etc. [14, 15]. With the further development of the disease, the intensification of oxidative stress reactions and the continuous destruction of microvascular permeability, the glomerular sclerosis speed is accelerated, and then it develops into a large amount of proteinuria, elevated blood creatinine, hypertension, and even uremia [16]. Therefore, early treatment of DM is of great significance.

The article "Effects of Shenkang Injection Combined with Jinshuibao on Early Diabetic Nephropathy and Effects on Coagulation Fibrinolysis System and Urinary Protein" was retracted in 2023. Reasons: signs of a paper mill; suspected computer-generated content; unreliable results or conclusions; concerns about the data.

DN belongs to the category of “oedema,” “deficiency labour,” and “thirst” in traditional Chinese medicine. The early stage of the disease is characterised by clear evidence of “stasis” and “deficiency.” Thus, the treatment of early DN focuses on controlling urine protein, improving kidney microcirculation (i.e., activating blood circulation and removing blood stasis), and nourishing kidney qi. SKI is composed of four herbs: rhubarb, *Astragalus* membranaceus, *Salvia miltiorrhiza,* and safflower. Among them, rhubarb can dredge the viscera, remove dirt, eliminate edema, reduce blood creatinine and urea nitrogen, and delay glomerular interstitial fibrosis [17]. *Astragalus* membranaceus can replenish qi and nourish blood, invigorate righteousness and eliminate pathogenic factors, nourish the heart and dredge the pulse, invigorate the spleen and diuresis, improve glucose metabolism, and expand renal blood vessels and cardiac blood vessels at the same time [18]. Pharmacological research [19] found that the main components of *Astragalus* membranaceus are astragalus polysaccharides, amino acids, linoleic acid, alkaloids, etc., which can enhance the immune function of the body, reduce the excretion of MA, and inhibit glomerular hypertrophy. At the same time, *Astragalus* can inhibit the production of transforming growth factor (TGF-B), reduce the level of vascular endothelin and the permeability of renal basement membrane so as to protect renal function and delay the deterioration of the renal function. When the two herbs mentioned above are used together, they both contribute to the improvement of gastrointestinal function. One falls and the other rises in their medicinal properties, dispelling turbidity, resolving stasis, and slowing down the deterioration of the kidney function. Both Salvia miltiorrhiza and safflower can activate blood circulation and improve blood circulation in the glomerulus. Animal experiments [20] showed that SKI could significantly reduce blood creatinine and urea nitrogen levels in 5/6 nephrectomized rats, reduce renal pathological damage, and lower urinary albumin, which may be the mechanism of its action to delay the progression of renal function deterioration. In addition, SKI has been shown to improve anaemia, increase plasma colloid osmotic pressure, raise plasma albumin, and reduce the amount of albumin in urine [21].

The main component of Jinshuibao is fermented Cordyceps powder. The adenosine, vitamin E, zinc, selenium, and copper contained in it directly participate in the metabolism of SOD, increase SOD, remove free radicals, reduce lipid peroxide, and protect the patient's kidney from damage. At the same time, it can improve renal blood flow, inhibit platelet aggregation, stabilize the lysosomal membrane, reduce NAG enzyme, maintain renal tubular function, reduce azotemia, protect and maintain renal function, and promote the repair of renal cells; and by regulating hormone secretion, it can enhance cellular immune function and phagocytosis of phagocytes, and play a certain role in the regulation and clearance of blood creatinine, urea nitrogen, and other metabolites. As a result, the internal environment of DN patients is brought from imbalance to balance, thus improving and stabilizing the condition, delaying the process of DN and renal insufficiency, reducing or decreasing the excretion of urinary protein, promoting the repair of renal tubular epithelial cells, inhibiting tubular atrophy and interstitial fibrosis, and achieving renal protection.

The article "Effects of Shenkang Injection Combined with Jinshuibao on Early Diabetic Nephropathy and Effects on Coagulation Fibrinolysis System and Urinary Protein" was retracted in 2023. Reasons: signs of a paper mill; suspected computer-generated content; unreliable results or conclusions; concerns about the data.

Several studies [22, 23] have shown that SKI plays an active role in activating blood circulation and removing blood stasis, improving hemodynamics, and reducing inflammatory reactions in the blood and urinary protein. Jinshuibao can regulate the expression level of signal pathway proteins in patients with DN, which not only has a good curative effect and reduces renal inflammatory reaction but also has the effect of nourishing the kidney [24, 25]. The results of this study show that after treatment, the observation group was more effective; the indexes related to urinary protein and coagulation and fibrinolysis for 2 groups were better than before, and the observation group changed significantly; there was no significant increase during the treatment in adverse reactions in the observation group. The results further showed that SKI in combination with Jinshuibao for early DN improved the coagulation and fibrinolysis system and did not significantly increase the incidence of adverse effects. The possible reasons for this are that early DN patients mostly have urinary protein, hypercoagulation, and fibrinogenic abnormalities. In this study, the application of SKI has obvious effects of dilating blood vessels, regulating blood lipids, reducing blood viscosity, and inhibiting platelet and red blood cell aggregation, thus increasing renal blood flow, reducing glomerular capillary pressure, improving glomerular blood hypercoagulation, and finally achieving the effect of reducing urinary protein; and the combination of Jinshuibao can further protect the kidney and regulate the oxidative stress response in the kidney so as to effectively improve the course of early DN.

The article "Effects of Shenkang Injection Combined with Jinshuibao on Early Diabetic Nephropathy and Effects on Coagulation Fibrinolysis System and Urinary Protein" was retracted in 2023. Reasons: signs of a paper mill; suspected computer-generated content; unreliable results or conclusions; concerns about the data.

In summary, SKI combined with Jinshuibao has a significant effect in the treatment of early DN, which can reduce the risk of hyperfunction of coagulation and fibrinolysis system, further reduce the content of urine protein, and delay the progression of renal disease in DM patients.

## Figures and Tables

**Figure 1:** Comparison of coagulation and fibrinolytic parameters for 2 groups (*n*, $\bar{x}\pm s$). Note: (a) PT (s). (b) APTT (s). (c) TT (s). (d) FIB (g/L). (e) PAI-1 (*μ*g/L). (f) t-PA (*μ*g/L). (g) D-D (*μ*g/L). ^*∗*^ and ^#^ represent comparison with the same group before treatment and comparison with the control group after treatment, respectively, *P* < 0.05.

**Figure 2:** Comparison of urine protein indicators for 2 groups (*n*, $\bar{x}\pm s$). Note: (a) 24 h-UTP (g/24 h). (b) UAER (*μ*g/min). (c) *β*2-MG (mg/L). ^*∗*^ and ^#^ represent comparison with the same group before treatment and comparison with the control group after treatment, respectively, *P* < 0.05.

**Table 1:** Comparison of post-treatment outcomes for 2 groups (*n*, %).

Group	*n*	Apparently cured	Improved	Invalid	Total effective
Control group	68	19 (27.94%)	35 (51.47%)	14 (20.59%)	54 (79.41%)
Observation group	68	25 (36.76%)	38 (55.88%)	5 (7.35%)	63 (92.65%)
*χ* ^2^ value					4.956
*P* value					0.026

## Data Availability

The data used or analysed during the study can be obtained from the corresponding author upon request.
